# Hepatic arterial infusion in combination with systemic chemotherapy in patients with hepatic metastasis from colorectal cancer: a randomized phase II study – (NCT05103020) – study protocol

**DOI:** 10.1186/s12885-023-11085-w

**Published:** 2023-07-22

**Authors:** Ji Su Kim, Hyunwook Kim, Seo Young Lee, Yoon Dae Han, Kichang Han, Byung Soh Min, Man-Deuk Kim, Jong Yun Won, Seung-Hoon Beom, Sang Joon Shin, Han Sang Kim, Dai Hoon Han, Joong Bae Ahn

**Affiliations:** 1 Division of Hepatobiliary and Pancreas Surgery, Incheon St. Mary’s Hospital, The Catholic University College of Medicine, Incheon, Korea; 2 Yonsei Cancer Center, Division of Medical Oncology, Department of Internal Medicine, Yonsei University College of Medicine, 50-1 Yonsei-Ro, Seodaemun-Gu, Seoul, 03722 South Korea; 3 Department of Medical Oncology, Gangnam Severance Hospital, Yonsei University College of Medicine, Seoul, Korea; 4 Department of Colorectal Surgery, Severance Hospital, Yonsei University College of Medicine, Seoul, Korea; 5 Department of Radiology, Severance Hospital, Yonsei University College of Medicine, Seoul, Korea; 6 Graduate School of Medical Science, Brain Korea 21 Project, Severance Biomedical Science Institute, Yonsei University College of Medicine, Seoul, South Korea; 7 Department of Hepatobiliary and Pancreatic Surgery, Severance Hospital, Yonsei University College of Medicine, 50 Yonsei-Ro, Seodaemun-Gu, Seoul, 03722 South Korea

**Keywords:** Colon cancer, Liver-only metastasis, Liver resection, Hepatic arterial infusion, Oxaliplatin, Randomized trial

## Abstract

**Background:**

Although 80% of patients with metastatic colorectal cancer (CRC) experience liver metastases, only 10–25% undergo resection at the time of diagnosis. Even in initially unresectable conditions, if appropriate treatment is provided, such as surgical conversion through a combination of hepatic arterial infusion (HAI) chemotherapy and systemic chemotherapy (sys-CT), better overall survival can be expected. Therefore, this study aims to evaluate the efficacy of HAI oxaliplatin in combination with sys-CT plus targeted therapy in patients with unresectable CRC with liver-only metastasis.

**Methods:**

This is a single-center, randomized, open-label phase II trial (NCT05103020). Patients with untreated CRC, who have liver-only metastases and for whom liver resection is potentially possible but deemed infeasible at the time of initial diagnosis by a multidisciplinary team, will be eligible. Patients will be randomly assigned in a 1:1 ratio to either the combined HAI oxaliplatin and modified systemic 5-fluorouracil, folinic acid, and irinotecan (FOLFIRI) plus targeted therapy group or the systemic FOLFIRI plus targeted therapy group. Both regimens will be repeated every 2 weeks for a total of 12 cycles. The primary objective of this study is to compare the rate of conversion to liver resection. The surgical conversion rate is expected to increase by 25% with HAI oxaliplatin in combination with sys-CT plus targeted therapy (40% in the experimental arm versus 15% in the control arm) (power, 80%; two-sided alpha-risk, 5%). The secondary objectives include overall survival, progression-free survival, and objective response rate.

**Discussion:**

This is the first randomized controlled trial to investigate the efficacy of HAI oxaliplatin in combination with sys-CT plus targeted therapy as first-line treatment from the initial diagnosis in patients with unresectable CRC with liver-only metastasis, aiming to significantly increase the surgical conversion rate.

**Trial registration:**

ClinicalTrials.gov, (NCT05103020). Trial registration date: November 2, 2021.

## Background

The liver is the most common site of metastasis in patients with colorectal cancer (CRC). Approximately 80% of patients with stage IV disease experience liver metastasis. Of these, approximately 40% experience metastasis that is only limited to the liver [1, 2]. However, only 15–25% of patients present with resectable colorectal liver metastasis (CRLM) at the time of diagnosis [3, 4]. If all liver metastases are completely resected, then the 5-year survival rate of these patients may exceed 50% [5, 6]. Furthermore, some patients may even be cured during the long-term follow-up, with a reported cure rate of approximately 20% [5].

### Conversion to surgery in patients with unresectable CRLM after systemic chemotherapy

Systemic chemotherapy (sys-CT) has been employed as neoadjuvant chemotherapy to help patients who cannot undergo liver resection at the time of diagnosis to become eligible candidates for surgery. According to a previous study, the surgical conversion rate ranges from 6 to 38%, depending on the type and duration of sys-CT and the anatomical extent of the liver metastases [7]. Several trials involving the combination of systemic chemotherapeutics with or without targeted therapies have demonstrated the downstaging of CRLM patients from initially inoperable to potentially resectable, and it was found that the objective response rate correlates with resectability [8–10]. R0 resection was possible in 19% of 196 patients with liver metastases of CRC, in whom liver resection is considered infeasible, following treatment with 5-fluorouracil (5-FU), leucovorin, oxaliplatin, and irinotecan (FOLFOXIRI). The median overall survival (OS) was 40 months, the 5-year disease-free survival rate was 29%, and the 5-year and 8-year survival rates were 42% and 33%, respectively [11].

### Hepatic arterial infusion chemotherapy

Hepatic arterial infusion (HAI) is a treatment method in which an interventional radiologist or surgeon inserts a port into the gastroduodenal artery, allowing direct delivery of anticancer therapeutics into the liver. Several studies have employed HAI to treat metastatic liver cancers because these lesions receive their primary vascular supply from the gastroduodenal artery. As most chemotherapeutic agents used in HAI undergo direct liver metabolism, they are expected to present a lower risk of systemic exposure and toxicity compared to those used in sys-CT protocols [12].

Fast-metabolized fluorodeoxyuridine (FUDR), 5-FU, mitomycin-C, and oxaliplatin are also being investigated for their potential use in the HAI technique [13–16]. FUDR has been widely investigated, but its routine implementation in clinical practice is hampered by certain constraints, such as the need for a 14-day continuous infusion via a pump and the inherent risk of biliary toxicity, which is unexpectedly increased with bevacizumab [17]. HAI oxaliplatin is known to accumulate in a higher concentration in liver metastases than in normal parenchyma [18], only requires a 2-h infusion time, and has a more favorable toxicity profile with reduced biliary toxicity. Moreover, even in later treatment stages, HAI oxaliplatin has shown a promising conversion rate of approximately 25%. Importantly, it has also proven effective in cases that showed resistance to systemic oxaliplatin [16, 19, 20]. Furthermore, HAI treatment is known to be more effective when the number of prior sys-CT lines are less than two [16, 21].

### Combined treatment with HAI chemotherapy and sys-CT

To maximize the efficacy of HAI chemotherapy, it is essential to find the optimal sys-CT combination. Previous studies have shown that the surgical conversion rate increased to 25–47% and OS improved when HAI and sys-CT were used in combination, even in patients initially diagnosed with unresectable conditions [22]. However, contrasting findings have also been reported [23, 24]. Therefore, additional prospective trials are necessary to clarify these discrepancies and establish more definitive guidelines for the use of HAI treatment. At present, the SULTAN-PRODIGE53 (NCT03164655), a randomized phase II study, is investigating the intensified treatment combination of HAI oxaliplatin and systemic FOLFIRI plus targeted therapy compared to sys-CT alone in CRLM patients who remain non-resectable after 2–6 months of first-line induction sys-CT [25].

In order to optimize the efficacy of HAI treatment and maximize the surgical conversion rate, it is essential to investigate the utility of HAI in conjunction with sys-CT, starting from the initial induction of chemotherapy. However, till date, no research has been conducted on this aspect. Therefore, this study aims to evaluate the concurrent use of HAI oxaliplatin and sys-CT at the time of initial diagnosis in patients with CRLM. The primary goal is to maximize the conversion rate to surgery in a shorter period with less systemic toxicity by comparing it with that of the existing irinotecan-based standard treatment.

## Methods/design

### Patients and study design

This study is designed as an open-label, single-center, randomized phase II clinical trial to compare and evaluate the efficacy of the combination of HAI oxaliplatin with sys-CT (FOLFIRI) plus targeted therapy (bevacizumab or cetuximab) in treatment-naive patients with CRC with potentially resectable liver-only metastases. The study flowchart is presented in Fig. 1.

**Fig. 1:** Flow diagram of the trial. A total of 108 treatment-naïve patients with colon cancer with liver-only metastasis will be randomized in a ratio of 1:1 to the HAI oxaliplatin combined with systemic modified FOLFIRI plus targeted therapy group, or the systemic FOLFIRI plus targeted therapy group. *HAI* Hepatic artery infusion, 5*-FU*: 5-fluorouracil, *CEA* Carcinoembryonic antigen, *CT* Computed tomography, *MRI* Magnetic resonance imaging, *FOLFIRI*: 5-fluorouracil, folinic acid and irinotecan, *ECOG* Eastern cooperative oncology group, *PS* Performance status

The eligibility criteria will be as follows: (1) patients aged at least 19 years, (2) Eastern Cooperative Oncology Group Performance Status (ECOG PS) 0 or 1, and (3) life expectancy of at least 3 months. Unsuitability for liver resection will be ascertained by a multidisciplinary team (surgeon, radiologist, interventional radiologist, and oncologist) based on criteria enumerated in Table 1. Patients will be assigned randomly at a central institution to one of the two arms in a 1:1 ratio using the stratified permuted block randomization approach, with the ECOG PS and prior adjuvant chemotherapy experience as the stratification factors, viz. 2-h HAI oxaliplatin 100 mg/m^2^ and a systemic modified FOLFIRI regimen (1.5-h intravenous irinotecan 180 mg/m^2^ on day 1, 2-h intravenous leucovorin 400 mg/m^2^ followed by 46-h intravenous 5-FU 2400 mg/m^2^ on day 1 without 5-FU bolus) plus targeted therapy (2-h intravenous cetuximab 500 mg/m^2^ or 30-min intravenous bevacizumab 5 mg/kg) (experimental arm), or systemic FOLFIRI (1.5-h intravenous irinotecan 180 mg/m^2^ on day 1, intravenous 5-FU bolus 400 mg/m^2^, and 2-h intravenous leucovorin 400 mg/m^2^ followed by 46-h intravenous 5-FU 2400 mg/m^2^ on day 1) plus targeted therapy (2-h IV cetuximab 500 mg/m^2^ or 30-min intravenous bevacizumab 5 mg/kg) (control arm). Both regimens will be repeated every 2 weeks for a total of at least 4 cycles, but no more than 12 cycles, depending on the circumstances. Treatment will continue until the cancer is deemed resectable, the cancer progresses, drug toxicity occurs, or the patient refuses further treatment. After 12 cycles, the decision will be made by the researcher on whether to proceed with surgery or to continue with palliative chemotherapy. For those in the experimental arm, 5-FU plus leucovorin is to be continued at least until disease progression, intolerable side effects, or patient withdrawal of consent, even if it is difficult to maintain the HAI treatment due to the side-effects.

**Table 1:** Key Inclusion and exclusion criteria

**Inclusion criteria**	
• Age ≥ 19 years	
• ECOG PS ≤ 1	
• Advanced colorectal cancer (stage IV) with histologically proven unresectable liver-only metastases	
• Evaluation of unresectable liver metastases based on imaging tests (CT/MRI) by a multidisciplinary team (including surgeons, radiologists, interventional radiologists, and medical oncologists)	
• Criteria for unresectability	
° Upfront R0/R1 resection of all CRLM (leaves at least two adequately perfused and drained segments) is not possible	
° And/or metastases in contact with major vessels of the remnant liver, which would require resection of the vessel for R0 resection (i.e., tumor involvement of the main right and left portal veins, three main hepatic veins, or retrohepatic vena cava)	
• No prior chemotherapy	
• Adequate organ function	
° ANC ≥ 1.5 × 10^9^/L	° Hb ≥ 9.0 g/dL (including transfusion)
° PLT ≥ 100 × 10^9^/L	° AST/ALT ≤ 5 × ULN, ALP ≤ 5 × ULN
° Total bilirubin ≤ 1.5 × ULN	° CrCl ≥ 45 mg/min (Cockcroft-Gault formula)
° Urine dipstick of proteinuria < 2 + (if ≥ 2 + , ≤ 1 g of protein/24 h)	
• Life expectancy ≥ 3 months	
**Exclusion criteria**	
• Anatomically or medically not suitable for complete surgical resection	
° Two or more tumors in all hepatic segments	
° Bilobar liver metastases and more than 3 lesions (> 3 cm) in the future remnant liver	
° Bilobar liver metastases and liver disease extending to > 50% of the organ	
• Extrahepatic metastasis	
• Peripheral neuropathy ≥ grade 2 (CTCAE ver.4.03)	
• Any other condition that may interfere with patients’ participation/evaluation in the study	

*ANC* Absolute neutrophil count, *Hb* Hemoglobin, *PLT* Platelet, *AST* Aspartate aminotransferase, *ALT* Alanine aminotransferase, *ALP* Alkaline phosphatase, *CrCl* Creatinine clearance, *CT* Computed tomography, *MRI* Magnetic resonance imaging, *ECOG* Eastern Cooperative Oncology Group, *PS* Performance status, *CRLM* Colorectal liver metastasis, *CTCAE* Common terminology criteria for adverse events, *ULN* Upper limit of normal

A HAI catheter will be implanted by an interventional radiologist. Access to the HAI catheter is restricted to medical professionals who are skilled in using the HAI catheter and are knowledgeable about and trained in HAI chemotherapy. Its condition and function will be examined before each use.

### Endpoints and assessments

The primary study objective is the rate of conversion to liver resection. The secondary objectives include OS, progression-free survival, and objective response rate.

Carcinoembryonic antigen testing, chest radiography, computed tomography/magnetic resonance imaging, and tumor assessment are to be conducted every 8 weeks. Follow-up will be conducted every 6 months for up to 4 years following randomization.

### Statistical considerations and analysis plan

We expect a gain of 25% of patients who will be converted to surgery from chemotherapy (40% in the experimental arm versus 15% in the control arm; power, 80%; two-sided alpha-risk, 5%). Overall, we aim to enroll a total of 108 participants (54 in each arm), assuming a drop-out rate of 10%.

A major statistical analysis of treatment efficacy will be performed on the intention-to-treat population. Categorical data will be summarized in tables showing the frequency and corresponding proportions for each treatment group. Serial data will be summarized by treatment group using frequency, mean, standard deviation, median (if applicable), minimum, and maximum values. The descriptive analysis will be summarized for each treatment group and as a whole, with a description of the characteristics of the pretreatment phase. Hazard ratio and 95% confidence interval will be calculated according to the Cox proportional-hazard model, and the survival curve will be calculated according to the Kaplan–Meier method. Safety will be assessed based on analysis of adverse events and findings from standard clinical routine laboratory testing.

### Toxicity monitoring

Clinical and laboratory adverse events/symptoms will be graded according to Common terminology criteria for adverse events version 4.03 [26]. Liver enzymes (alkaline phosphatase, aspartate aminotransferase, alanine aminotransferase, and bilirubin) will be closely monitored to evaluate liver and biliary toxicities. Once a dose reduction is made, no subsequent dose increase is permitted. However, if it is determined that the toxicity is related to the test drug, the investigator may reduce or discontinue the test drug at the discretion of the investigator by referring to the dose adjustment recommendation.

Granulocyte colony stimulating factor is not recommended as a primary prophylaxis. However, it can be used for secondary prevention in cases of prior febrile neutropenia, grade 4 neutropenia lasting for more than 5 days, or if the planned treatment is delayed by two or more times due to neutropenia.

If a patient undergoing HAI oxaliplatin treatment reports abdominal pain or catheter-related discomfort, it would be necessary to inspect the HAI catheter for potential issues, such as malfunction, infection, or leakage. If such problems are identified, the investigator should consider removing and reinserting the catheter at his or her discretion.

### Ancillary study: biomarker analysis

Transitional research investigates the correlation between the maximum tumor shrinkage rate and the variation of circulating tumor DNA (ctDNA) concentration, pre- and post-planned treatment. The relationship between the changes in circulating tumor cells and progression-free survival will also be explored. In addition, the concordance rate of mutation identification in formalin-fixed paraffin-embedded samples and ctDNA will be compared and assessed to discover KRAS exon 2 (G12X, G13X), exon 3 (Q61X), NRAS exon 2 (G12X), exon 3 (Q61X), and BRAF exon 15 (V600E) mutations.

### Data collection, management, and monitoring

All trial data will be collected and managed in papers and also maintained and monitored by the principal investigator at Yonsei Cancer Center. We estimated the patient accrual and study duration to take 2 and 4 years, respectively.

## Discussion

R0 resection is critical for the long-term survival of patients with stage IV CRC. Considering this might be the patient's last opportunity for a cure, finding a more effective treatment strategy is crucial. Such a strategy could allow curative aim surgery to be performed on patients initially considered unsuitable for liver resection at diagnosis. The group treated with systemic bevacizumab-FOLFOXIRI in the OLIVIA trial [9] not only demonstrated higher response rates, but also a higher resection rate of 61% (95% CI, 45–76%) and an R0 resection rate of 49% when compared to those of the bevacizumab-mFOLFOX-6 group. However, more than 95% of patients experienced toxicity events of grade 3 or higher. As a result, there is an urgent need to continue efforts to develop more tolerable and safer treatment methods. In this regard, the therapeutic regimen of HAI oxaliplatin combined with modified FOLFIRI plus targeted therapy is thought to reflect these requirements well. However, there are also several limitations to consider. To administer HAI chemotherapy, an invasive procedure for the insertion of an intra-arterial port is necessary. There is also a risk of liver injury due to the HAI catheter tip, which requires caution. Moreover, the complexity of these procedures makes widespread adoption across all institutions difficult.

Another important point in this study is the need to determine the possibility of liver resection in a timely manner while receiving systemic treatment. A multidisciplinary approach is required to evaluate the likelihood of resection, taking into account the condition of the tumor before and after chemotherapy, as well as the performance status of the patient, environment, and life expectancy. To conduct this evaluation in a comprehensive manner, surgeons, radiologists, and physicians should jointly review every radiologic image for response evaluation. Most importantly, the surgeon's perspective is particularly significant in this context.

This is the first randomized controlled trial to investigate HAI oxaliplatin in combination with sys-CT plus targeted therapy as first-line treatment from the initial diagnosis in patients with CRC with potentially resectable liver-only metastasis.The primary objective of this trial is to significantly increase the surgical conversion rate. We plan to include 108 patients, and the recruitment period and observation period are 2 years each. While direct comparison with the ongoing SULTAN-PRODIGE53 study (NCT03164655) [16] is challenging, the results from both studies will provide valuable insights into the role and optimal application timing of HAI treatments. Further research is necessary to determine which patients will benefit the most from HAI combination, as well as to ascertain the optimal sys-CT and targeted agent combination regimen and the ideal duration of post-operative systemic therapy for maintaining a disease-free status.

## Data Availability

Not applicable.

## Abbreviations

CRC: Colorectal cancer
HAI: Hepatic arterial infusion
5-FU: 5-Fluorouracil
CRLM: Colorectal liver metastasis
ctDNA: Circulating tumor DNA
ECOG: Eastern cooperative oncology group
PS: Performance status
FOLFIRI: 5-Fluorouracil, folinic acid, and irinotecan
FUDR: Fluorodeoxyuridine
OS: Overall survival
sys-CT: Systemic chemotherapy
FOLFOXIRI: 5-Fluorouracil, leucovorin, oxaliplatin, and irinotecan
